The article "Diagnosis of Lofgren’s Syndrome and the Role of Ultrasound" was published in 2021. Journal: Cureus.

# Diagnosis of Lofgren’s Syndrome and the Role of Ultrasound

**DOI:** 10.7759/cureus.20332

**Published:** 2021-12-10

**Authors:** Rita Costa, Nuno Leal, Pedro Salvador, Pedro Oliveira, Carina Silva

**Affiliations:** 1 Internal Medicine, Centro Hospitalar Vila Nova de Gaia/Espinho, Vila Nova de Gaia, PRT

**Keywords:** ultrasound, arthralgia, erythema nodosum, mediastinal lymphadenopathy, sarcoidosis, loefgren

## Abstract

We report the case of a 32-year-old woman presenting to the emergency department with ankle edema and arthralgia. Only later in the follow-up period, she developed erythema nodosum. The study revealed bilateral hilar and mediastinal lymphadenopathy and biopsy demonstrated non-caseating granulomas consistent with a diagnosis of Lofgren’s syndrome. Patients often do not present with all signs and symptoms, which delays the correct diagnosis. This case reinforces the need to use diagnostic methods, particularly non-invasive ones, such as ultrasound (US), in such cases. US of the lower extremity swelling could have helped the diagnosis, even without demonstrating effusion.

## Introduction

Sarcoidosis is a chronic multisystem granulomatous inflammatory disorder, whose etiology is not fully understood and the diagnosis can be challenging [1]. Rarely does the patient present with a “full picture”; furthermore, different conditions have similar manifestations and there is no definitive diagnostic test. Lofgren’s syndrome is an acute form of sarcoidosis and is defined by the triad erythema nodosum, hilar pulmonary adenopathy and arthralgia [2].

Arthritis involves preferentially the ankles, and it is often the initial feature of sarcoidosis [3,4]. Tenosynovitis with periarticular edema and subcutaneous or periarticular inflammation is part of the spectrum of articular manifestations of sarcoidosis [3,5]. Ultrasound (US) is more sensitive in identifying these changes and acts as a simple, economical, innocuous diagnostic method that could shorten the diagnosis. Lofgren’s syndrome usually has a good prognosis. The course of the disease is mostly self-limited and responds to non-steroidal anti-inflammatory drugs (NSAIDs).

## Case presentation

A 32-year-old woman, with no previous relevant clinical history, was admitted to the emergency room in August 2020 with complaints of significant arthralgia and ankle edema. She mentioned a progressive evolution with additive joint disease in the previous week, now involving ankles, knees, wrist and proximal interphalangeal and metacarpophalangeal joints. The initial physical examination showed no fever, mild swelling and tenderness in both ankles, without limitation of range of motion. At admission, she presented with no other signs of arthritis, but the pain was now present, limiting the ability of performing the daily living activities despite the use of NSAIDs. She was discharged to an early appointment to follow up. Later she developed painful erythematous nodules below the knees and pretibial localization.

The article "Diagnosis of Lofgren’s Syndrome and the Role of Ultrasound" was published in 2021. Journal: Cureus.

Laboratory studies showed mild anemia (hemoglobin 11.7 g/dL), normal white blood cell count, but elevated erythrocyte sedimentation rate and C-reactive protein level (Table 1). Aspartate aminotransferase and alanine transaminase levels were normal. Renal function, calcium level (9.7 mg/dL) and remaining ionograms were normal. The serum angiotensin-converting enzyme (ACE) level was elevated. Rheumatoid factor and anti-cyclic citrullinated peptide (anti-CCP) antibody levels were both negative, complement levels were normal, antinuclear antibody was negative, and specific antibodies were not detected. Human immunodeficiency virus, syphilis and hepatitis B and C viruses were also excluded. Despite the visible edema and pain, the ankle US was innocent.

**Table 1:** Analytical data Ab: antibody; ELISA: enzyme-linked immunosorbent assay; PCR: polymerase chain reaction; PPD: purified protein derivative; RPR: rapid plasma regain; ACE, angiotensin-converting enzyme; IGRA, interferon-gamma release assay

Paraclinical test	Result	Reference interval
Serum calcium (mg/dL)	9.7	8.8-10.2
Antinuclear Ab (ANA)	Negative	–
Ab to extractable nuclear antigens	Negative	–
Antineutrophil cytoplasmic Ab cytoplasmic pattern (cANCA)	Negative	–
Antineutrophil cytoplasmic Ab perinuclear pattern (pANCA)	Negative	–
Complement fraction C3 (mg/dL)	181	77-135
Complement fraction C4 (mg/dL)	20.9	9-36
Rheumatoid factor (IU/mL)	<9.69	0-5.9
ACE (U/L)	70	8-52
Human immunodeficiency virus types 1 and 2 (ELISA)	0.1 (non-reactive)	>1.1 reactive
Syphilis (RPR)	Non-reactive	–
Mycobacterium tuberculosis (bronchoalveolar lavage - PCR and cultural)	Negative	
IGRA	Negative	
Antibody against hepatitis C virus	0.05 (non-reactive)	>1.1 reactive
Hepatitis B virus surface antigen	0.2 (non-reactive)	>1.1 reactive
C-reactive protein (mg/dL)	9	0-0.5
Erythrocyte sedimentation rate (mm/h)	47	0-15

The chest X-ray demonstrated mediastinal widening. She then underwent a chest computed tomography (CT) scan that demonstrated numerous peritracheal and hilar adenomegaly with numerous, predominantly peripheral subpleural or pericissural, nodules, compatible with sarcoidosis (Figure 1). The patient underwent endobronchial ultrasound bronchoscopy and the biopsy demonstrated epithelioid granulomas with multinucleated giant cells, without necrosis. Bronchoalveolar lavage fluid revealed an elevated total cell count, predominantly lymphocytes, elevated CD4/CD8 ratio, and a nearly normal percentage of eosinophils and polymorphonuclear neutrophils.

The article "Diagnosis of Lofgren’s Syndrome and the Role of Ultrasound" was published in 2021. Journal: Cureus.

**Figure 1:** Chest CT scan showing bilateral hilar mediastinal adenopathy marked with a red circle

Thus, the triad of acute polyarthritis, hilar adenopathy and erythema nodosum, reinforced with the biopsy results, led to the diagnosis of Lofgren's syndrome.

In our patient, the symptoms were very debilitating even with using analgesics such as paracetamol and NSAIDs. Therefore, in order to reduce inflammation and control symptoms, the patient did a short course of corticosteroids.

## Discussion

Intrathoracic involvement is the hallmark of sarcoidosis, present in over 90% of patients [2,6]. Notwithstanding, it also commonly affects the skin [2,7].

Lofgren’s syndrome was first described by a Swedish pulmonologist, Sven Lofgren, in 1952 [2]. The peak incidence occurs between 30 and 40 years of age and women seem to be more affected and have a second peak between 45 and 65 years of age [2,8]. Lofgren’s syndrome has a clinically distinct phenotype. It usually presents acutely, with erythema nodosum, bilateral hilar lymphadenopathy, and the presence of arthritis/arthralgia [2,8]. In contrast, sarcoidosis usually has an insidious onset and a slow progression to chronic disease.

The anamnesis and thoracic imaging are essential for the diagnosis, although tissue biopsy demonstrating the non-caseating granulomas is needed for a definitive diagnosis [9]. Other granulomatous diseases mimicking sarcoidosis, such as tuberculosis, must be excluded. Histological confirmation is not needed for Lofgren’s syndrome.

An important detail of the reported case is the fact that the patient presented initially with periarticular ankle inflammation and edema without apparent arthritis or erythema nodosum. This periarticular inflammation has been previously mentioned as a variant of the Lofgren’s syndrome [3,10]. It usually presents as an association with bilateral hilar adenopathy and usually follows a benign course to total remission. Besides, it has been proven in previous studies that ankle involvement in patients with Lofgren’s syndrome is more frequently periarticular rather than articular [10]. In these patients, musculoskeletal US could be a first-line diagnostic exam. US in Lofgren’s syndrome cases usually shows hypervascular subcutaneous edema (82%-92%) and tenosynovitis (33%-39%) [3,11]. If this entity was part of the differential diagnosis of patients with distal lower extremity swelling, with trained radiologists, the diagnosis could be shortened with this non-invasive and radiation-free exam [11].

## Conclusions

This report aims to highlight an uncommon disease Lofgren’s syndrome, focusing on the diagnosis of this rare condition. We would like to emphasize the potential of musculoskeletal US in the diagnosis of this rheumatologic disease. If this entity is considered in the differential diagnosis of lower extremity swelling and tenosynovitis of the ankle, even without clear signs of joint effusion, it could narrow down the diagnosis.
